# An Online Weighted Bayesian Fuzzy Clustering Method for Large Medical Data Sets

**DOI:** 10.1155/2022/6168785

**Published:** 2022-02-21

**Authors:** Cong Zhang, Jing Xue, Xiaoqing Gu

**Affiliations:** ^1^School of Computer and Information Engineering, Nantong Polytechnic College, Nantong 226001, Jiangsu, China; ^2^Department of Nephrology, The Affiliated Wuxi People's Hospital of Nanjing Medical University, Wuxi 214023, Jiangsu, China; ^3^School of Computer Science and Artificial Intelligence, Changzhou University, Changzhou, 213164, Jiangsu, China

## Abstract

With the rapid development of artificial intelligence, various medical devices and wearable devices have emerged, enabling people to collect various health data of themselves in hospitals or other places. This has led to a substantial increase in the scale of medical data, and it is impossible to import these data into memory at one time. As a result, the hardware requirements of the computer become higher and the time consumption increases. This paper introduces an online clustering framework, divides the large data set into several small data blocks, processes each data block by weighting clustering, and obtains the cluster center and corresponding weight of each data block. Finally, the final cluster center is obtained by processing these cluster centers and corresponding weights, so as to accelerate clustering processing and reduce memory consumption. Extensive experiments are performed on UCI standard database, real cancer data set, and brain CT image data set. The experimental results show that the proposed method is superior to previous methods in less time consumption and good clustering performance.

## 1. Introduction

In recent years, smart medical care has emerged with the vigorous development of artificial intelligence (AI) technology. At present, the application of AI technology in the medical field involves many aspects such as disease prediction, intervention and consultation, disease diagnosis and treatment, drug research and development, and health service management [1]. The fusion of AI and healthcare services can help clinicians reduce reading time, aid in early detection, and improve diagnostic accuracy. The technology of clustering plays a very wide role in the fields of medical data analysis.

As a typical unsupervised learning method, clustering mines the internal relationship between data samples and then puts the samples with the same or similar attributes in the same cluster, which avoids the dependence on the label data and saves a lot of manpower and material resources [2]. Fuzzy clustering is a typical representative of clustering methods, and the most classic fuzzy clustering is the fuzzy *C*-means algorithm (FCM). Fuzzy clustering improves the traditional hard clustering partition. There are a large number of derivative algorithms based on the FCM, including the probabilistic *C*-means algorithm (PCM), which uses probabilistic methods to express fuzzy membership to improve the limitation of fuzzy membership [3]. Recently, many researchers have improved the traditional FCM method from multiple perspectives and applied them in various scenes [4]. Hua et al. [5] developed a multiview fuzzy clustering based on the framework of FCM. Gu et al. [6] proposed a probabilistic FCM method to be used for antecedent parameter learning in Takagi-Sugeno-Kang fuzzy system. Zhou et al. [7] proposed a new membership scaling FCM method by selecting the unchanged clustering centers through triangular inequality, which solves the problems of slow convergence and a large amount of calculation when a FCM algorithm is dealing with large data sets. Mishro et al. [8] proposed a new type 2 adaptive weighted space FCM clustering algorithm to solve the problem of noise misclassification and inaccurate clustering center obtained by FCM in the process of MR brain image segmentation. Wang et al. [9] proposed an FCM algorithm for irregular image segmentation, which has higher robustness and less computational effort compared to traditional segmentation algorithms. Based on hyperplane partitioning, Shen et al. [10] developed a feasible and efficient FCM algorithm to deal with large data sets. Jha et al. [11] designed and implemented a kernelized fuzzy clustering algorithm using its in-memory cluster computing technology. Liu et al. [12] proposed a FCM algorithm based on multiple surface approximate interval membership for processing artifacts in brain MRI images. Wang et al. [13] proposed a FCM algorithm based on wavelet frame, which can effectively remove image noise and preserve image details. This algorithm can provide a new way to segment images in an irregular domain. Li et al. [14] proposed a domain-qualified adaptive FCM method for processing MRI brain images with noise and uneven intensity. Zhang and Huang [15] studied the generalization error of a FCM algorithm from the perspective of theory and limited the generalization error from the perspective of convergence, which can provide guidance for the application of the sampling-based FCM method. Wu et al. [16] proposed an online clustering algorithm by combining FCM algorithm with an online framework set to solve the problem that batch learning cannot deal with large-scale data sets. Zhang et al. [17] combined FCM with a nonlinear genetic algorithm and proposed an apple defect detection method to improve fruit defect detection. Shen et al. [18] proposed a hyperplane partition method based on FCM to deal with big data clustering. Recently, the Bayesian fuzzy clustering (BFC) [19] algorithm is proposed to combine the fuzzy method into a probability model. BFC reinterprets the fuzzy method from the perspective of probability, expands the value range of the fuzzy index, and solves the problem that the fuzzy method is prone to local optimization. The many characteristics of the BFC algorithm make it very widely used in medical data processing. But due to the high complexity of the BFC method, its efficiency is not high, and it has received great limitations in practical applications.

Inspired by the above ideas, this paper proposes the online weighted Bayesian fuzzy clustering method (OWBFC) and uses an online clustering framework, which not only retains all the advantages of the Bayesian fuzzy clustering algorithm but also improves the efficiency of the Bayesian fuzzy clustering method through the online clustering framework. We verify the OWBFC method on a series of real-world data sets. Compared with the existed Bayesian fuzzy clustering algorithms, the contributions of our study are concluded as follows:

1. OWBFC combines the probability method with the fuzzy method and realizes the fuzzy clustering through the probability method, which has the common advantages of the probability method and the fuzzy method.
2. In the process of solving the parameters, the Markov chain Monte Carlo method (MCMC) is used for sampling instead of a closed solution, so the global optimal solution of the parameters can be obtained in OWBFC.
3. The online clustering framework is used in OWBFC to deal with the problem that large data sets cannot be imported into memory, and the weighting mechanism is used to improve the clustering efficiency.

## 2. Related Work

The BFC algorithm combines the probabilistic method with the fuzzy method. From the perspective of prior knowledge and Bayesian theory, it expands the range of the fuzzy index of the traditional fuzzy method. The BFC algorithm uses the MCMC strategy [20] and particle filter method [21, 22] to solve the optimization problem. The maximum posterior probability (MAP) is used to process fuzzy clustering, and the normal distribution is further used to predict the number of clusters. Therefore, the BFC method is superior to the previous fuzzy or probabilistic methods in many aspects. However, the algorithm complexity of BFC is relatively high. This shortcoming makes the BFC method not suitable for large-scale data, and its application range is greatly limited, which does not meet the current actual needs. The BFC algorithm aims to solve fuzzy clustering from the perspective of probability. The probability model of BFC consists of three parts, namely fuzzy data likelihood (FDL), fuzzy membership prior (FCP), and cluster center prior, as follows. The fuzzy data likelihood is as follows:

(1) $$\begin{array}{c} p\left(X\;|\;U,C\right)=\overset{K}{\underset{k=1}{\prod }}\mathrm{FDL}\left(x_{k}\;|\;u_{k},C\right)\\ =\overset{K}{\underset{k=1}{\prod }}\frac{1}{Z\left(u_{k},m,C\right)}\overset{N}{\underset{n=1}{\prod }}N\left(x_{k}\;|\;\mu =c_{n},\Lambda =u_{kn}^{m}I\right), \end{array}$$

where ***X***, ***U***, and ***C*** are matrices of training data, fuzzy member, and cluster centers, respectively. *K* and *N* represent the numbers of samples and the numbers of clusters, respectively. *u*_*kn*_ is the membership of data point **x**_*k*_ in cluster *n*. The parameters *m*, **c**_*n*_, and ***I*** represent the fuzzy index, the cluster center, and the identity matrix, respectively. And, *Z*(**u**_*k*_, *m*, **C**) is the normalization constant, and *m* is the fuzzy index. Since *Z*(**u**_*k*_, *m*, **C**) will be eliminated by the following equation (2), it does not need to be calculated.

The prior of fuzzy membership is expressed as

(2) $$\begin{array}{c} p\left(U|C\right)=\overset{K}{\underset{k=1}{\prod }}\mathrm{FCP}\left(u_{n}|C\right)\\ =\overset{K}{\underset{k=1}{\prod }}Z\left(u_{k},m,C\right)\left(\overset{N}{\underset{n=1}{\prod }}u_{kn}^{-m\;D/2}\right)\text{Dirichlet}\left(u_{k}|\alpha \right). \end{array}$$

*p*(**U***| ***C**) consists of three parts as follows: *F*_1_=*Z*(**u**_*k*_, *m*, **C**), *F*_2_=∏_*n*=1_^*N*^*u*_*kn*_^−*m*  *D*/2^, and *F*_3_=Dirichlet(**u**_*k*_*|α*). *F*_1_ is to eliminate the normalizing constant in equation (1). *F*_3_ is the Dirichlet distribution as follows:

(3) $$\begin{array}{c} \text{Dirichlet}\left(x|\alpha \right)=\frac{\Gamma \left(\sum_{n=1}^{N}\alpha_{n}\right)}{\prod_{n=1}^{N}\Gamma \left(\alpha_{n}\right)}\overset{N}{\underset{n=1}{\prod }}x_{n}^{\alpha_{n}-1}, \end{array}$$

where *x*_*n*_ ≥ 0, *n* = 1,…, *N* and ∑_*n*=1_^*N*^*x*_*n*_=1. The parameter *α* is the Dirichlet prior parameter, which controls the membership degree of the sample. Through Dirichlet distribution, the BFC algorithm breaks the constraint that the fuzzy index in the FCM algorithm must be greater than 1, so that the fuzzy index in the BFC algorithm can take any value.

Cluster center prior is defined as

(4) $$\begin{array}{c} p\left(C\right)=\overset{N}{\underset{n=1}{\prod }}N\left(c_{n}|\mu_{c},\Sigma_{c}\right). \end{array}$$

It is noted that *p*(**C**) is to match the high degree of membership produced by equation (4). *μ*_*c*_ and Σ_c_ are the mean and variance of all samples, as follows:

(5) $$\begin{array}{c} \mu_{c}=\frac{1}{K}\overset{K}{\underset{k=1}{\sum }}x_{k}\\ \Sigma_{c}=\frac{\gamma }{K}\overset{K}{\underset{k=1}{\sum }}\left(x_{k}-\mu_{c}\right){\left(x_{k}-\mu_{c}\right)}^{T}, \end{array}$$

where *γ* is a parameter that affects the strength of the prior, which is set by the user, and we use *γ* = 3 in our study. The joint likelihood of **X**, **U**, and **C** is obtained by multiplying equations (1), (2), and (4).

(6) $$\begin{array}{c} p\left(X,U,C\right)=p\left(X|U,C\right)p\left(U|C\right)p\left(C\right)\\ \propto exp\left\{-\frac{1}{2}\overset{K}{\underset{k=1}{\sum }}\overset{N}{\underset{n=1}{\sum }}u_{kn}^{m}||x_{k}-c_{n}|{|}^{2}\right\}\times \left[\overset{K}{\underset{k=1}{\prod }}\overset{N}{\underset{n=1}{\prod }}u_{kn}^{\alpha_{n}-1}\times \;\exp\left\{-\frac{1}{2}\overset{N}{\underset{n=1}{\sum }}{\left(c_{n}-\mu_{c}\right)}^{T}\overset{-1}{\underset{c}{\sum }}\left(c_{n}-\mu_{c}\right)\right\}\right]. \end{array}$$

According to map theory, the joint likelihood form of equation (7) is its negative logarithm, and a factor of 2 can be multiplied to simplify. The joint likelihood form is as follows:

(7) $$\begin{array}{c} J\left(X,U,C\right)=\overset{K}{\underset{k=1}{\sum }}\overset{N}{\underset{n=1}{\sum }}u_{kn}^{m}||x_{k}-c_{n}|{|}^{2}-2\overset{K}{\underset{k=1}{\sum }}\overset{N}{\underset{n=1}{\sum }}\left(\alpha_{n}-1\right)\text{log}u_{kn}+\overset{N}{\underset{n=1}{\sum }}{\left(c_{n}-\mu_{c}\right)}^{T}\overset{-1}{\underset{c}{\sum }}\left(c_{n}-\mu_{c}\right). \end{array}$$

Finally, BFC uses MAP inference and uses sampling to filter membership and cluster centers to obtain their optimal values.

From the above introduction, we can see that the BFC algorithm breaks through the constraints of the traditional fuzzy clustering fuzzy index and can obtain the global optimal solution, but its time complexity is too high to handle large data sets.

## 3. Online Weighted Bayesian Fuzzy Clustering

### 3.1. Weighted Bayesian Fuzzy Clustering

For large data sets, it is a difficult problem that the data cannot be imported into the computer at one time. In this paper, the online clustering framework is adopted. By dividing the large data set into several easy-to-handle small data blocks, the clustering center of each data block is defined as the representative point. In the process of processing the data blocks, the representative points of each data block and the corresponding weights of the representative points are combined into two new different sets, and then, the two new sets are processed to get the clustering center of the whole data and accelerate clustering. Since the OWBFC method uses a block and weighting mechanism to introduce weights for the clustering centers of each data block, the weighted Bayesian fuzzy clustering (WBFC) algorithm is introduced, and then, WBFC is extended to its online version.

To further judge the contribution of each sample point to the cluster in the process of clustering, this paper introduces the WBFC algorithm, which adaptively weights different sample points to select the representative sample points. The objective function of WBFC is defined as

(8) $$\begin{array}{c} p\left(X,U,C\right)=p\left(X|U,C\right)p\left(U|C\right)p\left(C\right)\\ \propto exp\left\{-\frac{1}{2}\overset{K}{\underset{k=1}{\sum }}\overset{N}{\underset{n=1}{\sum }}w_{n}u_{kn}^{m}||x_{k}-c_{n}|{|}^{2}\right\}\times \left[\overset{K}{\underset{k=1}{\prod }}\overset{N}{\underset{n=1}{\prod }}u_{kn}^{\alpha_{n}-1}\times \;\exp\left\{-\frac{1}{2}\overset{N}{\underset{n=1}{\sum }}{\left(c_{n}-\mu_{c}\right)}^{T}\overset{-1}{\underset{c}{\sum }}\left(c_{n}-\mu_{c}\right)\right\}\right], \end{array}$$

where *w*_*k*_ > 0 represents the contribution of the *n*th sample to the final cluster division. How to set *w*_*k*_ will be described in detail in the next section. Following [19], the MCMC parameter optimization strategy is used in the WBFC algorithm. First, we initialize the parameter **u**_*k*_ and **c**_*n*_ by Dirichlet distribution and normal distribution. We sample the ***U*** matrix according to **U** ~ *p*(**U***| ***X**, **C**) ∝ *p*(**X**, **U**, **C**) using the Gibbs sampling. We judge whether the new membership sample is accepted. If it is accepted, then **u**_*k*_ is set as **u**_*k*_=**u**_*k*_^Ψ^, **u**_*k*_^Ψ^ as a new membership sample. The acceptation rate *A*_**u**_ is computed as

(9) $$\begin{array}{c} A_{u}=\text{min}\left\{1,\frac{p\left(x_{k},u_{k}^{\Psi }|C\right)}{p\left(x_{k},u_{k}|C\right)}\right\}. \end{array}$$

If *p*(**x**_*k*_, **u**_*k*_^Ψ^*| ***C**^*∗*^) > *p*(**x**_*k*_, **u**_*k*_^*∗*^*| ***C**^*∗*^), we set the current **u**_*k*_^*∗*^ as **u**_*k*_^*∗*^=**u**_*k*_^Ψ^. The *p*(**x**_*k*_, **u**_*k*_*| ***C**) is computed as

(10) $$\begin{array}{c} p\left(x_{k},u_{k}|C\right)=p\left(x_{k}|u_{k},C\right)p\left(u_{k}|C\right)\propto \overset{N}{\underset{n=1}{\prod }}\exp\left(-\frac{1}{2}w_{k}u_{kn}^{m}{\left\|x_{k}-c_{n}\right\|}^{2}\right)u_{kn}^{\alpha_{n}-1}. \end{array}$$

Then, we sample ***C*** according to **C** ~ *p*(**C***| ***X**, **U**) ∝ *p*(**X**, **U**, **C**). We judge whether the new cluster center sample is accepted. If it is accepted, then **c**_*n*_ is set as **c**_*n*_=**c**_*n*_^Ψ^. The acceptation rate *A*_**c**_ is computed as

(11) $$\begin{array}{c} A_{c}=\min\left\{1,\frac{p\left(x_{k},c_{k}^{\Psi }|C\right)}{p\left(x_{k},c_{k}|C\right)}\right\}. \end{array}$$

If *p*(**X**, **c**_*n*_^Ψ^*| ***U**^*∗*^) > *p*(**X**, **c**_*n*_^*∗*^*| ***U**^*∗*^), we set the current **c**_*n*_^*∗*^ as **c**_*n*_^*∗*^=**c**_*n*_^Ψ^, **c**_*n*_^Ψ^ as a new cluster center. The *p*(**X**, **c**_*n*_*| ***U**) is computed as

(12) $$\begin{array}{c} p\left(X,c_{n}|U\right)=p\left(X|U,c_{n}\right)p\left(c_{n}\right)\propto exp\left\{-\frac{1}{2}\overset{K}{\underset{k=1}{\sum }}\overset{N}{\underset{n=1}{\sum }}w_{k}u_{kn}^{m}||x_{k}-c_{n}|{|}^{2}\right\}\times \;\exp\left\{-\frac{1}{2}\overset{N}{\underset{n=1}{\sum }}{\left(c_{n}-\mu_{c}\right)}^{T}\overset{-1}{\underset{c}{\sum }}\left(c_{n}-\mu_{c}\right)\right\}. \end{array}$$

Finally, we check the maximum likelihood of all samples using equation (9). The whole training process circulates several times until the model converges. The training procedure of WBFC is shown in Algorithm 1.

### 3.2. Online Weighted Bayesian Fuzzy Clustering

The WBFC algorithm aims to introduce object weights based on the BFC algorithm, so more representative sample points can be selected while clustering. Based on the characteristics of the WBFC algorithm, we further proposed the online version of WBFC algorithm called OWBFC algorithm. Inspired of the online algorithm advantage, the OWBFC algorithm can handle large data sets based on the WBFC algorithm. OWBFC divides the large-scale data into several easy-to-process data blocks. Then, OWBFC uses the WBFC algorithm to process each data block, merges the cluster center of each data block into a new set, calculates the weight of each cluster center, and merges the obtained weight. Finally, the new cluster center set and the corresponding weight set are processed to obtain the final cluster center. The weight factor *w*_*n*_ in OWBFC is computed as follows:

(13) $$\begin{array}{c} w_{q}=\overset{K_{l}}{\underset{k=1}{\sum }}u_{kq},q=1,\ldots ,\mathrm{Q,} \end{array}$$

where *w*_*q*_ represents the weight of representative points of each data block. Here, we give the training procedure of the OWBFC algorithm as shown in Algorithm 2. The parameter *K*_*l*_ represents the number of sample points in the *l*th block, *u*_*kq*_ is the membership of **x**_*k*_ in cluster *q*, and *Q* represents the number of clusters. First, we divide the training data ***X*** into *d* blocks as **X**={**X**_1_,…,**X**_*d*_}, and each block **X**_*l*_ has *K*_*l*_ sample points, *l* = 1, 2, ..., *d*. **U**_*l*_ and **C**_*l*_ are the fuzzy membership and clustering center matrices, respectively. We run the WBFC algorithm in the first block **X**_1_ and obtain the fuzzy membership and clustering center matrices in **X**_1_. Then, we run the WBFC algorithm in the rest blocks with the clustering center matrix ***C***_*l*-1_.

## 4. Experiments

### 4.1. Data Sets and Experiment Settings

In the experiment, we use several medical data sets, including two cancer data sets, Armstrong-2002-v2 and Bhattacharjee-2001 [23], three medical data sets, and brain images in the UCI database [24]. Armstrong-2002-v2 is a data set to distinguish the expression of leukemia genes. It is divided into three categories, with a total of 72 samples. Bhattacharjee-2001 is a lung cancer classification data set, including five categories, a total of 203 samples. Because of the small sample size of these two data sets, they are not segmented here. The heart disease data set, diabetic retinopathy Debrecen (DRD) data set, and hepatitis C virus (HCV) for Egyptian patient data set are three UCI medical data sets. The heart disease data set contains 303 samples, and only 14 of them are used in this article. The DRD data set contains 1151 samples, and the HCV data set contains 1385 samples. To facilitate the division, this study takes 1000 samples for the diabetic retinopathy Debrecen data set. The HCV data set took 1,200 samples. A total of three brain CT images were selected as CT1, CT2, and CT3, with pixels of 275 × 273, 273×277, and 264 × 271. To facilitate segmentation, the pixels of the three pictures are reduced to 272 × 272, 272 × 272, and 264 × 264, respectively. The comparison algorithms include OFCM [25] and SPFCM [25], which can process large-scale data clustering. Among them, the two cancer data sets and one UCI medical data set are used to compare the clustering effects of OWBFC, OFCM, and SPFCM algorithms without segmentation. The remaining two UCI medical data sets are used to compare the clustering effects and time of OWBFC, OFCM, and SPFCM algorithms in different proportions of segmentation. The brain images are used to show the running time comparison of OWBFC and BFC. The OWBFC, OFCM, and SPFCM algorithms have two parameters: fuzzy index *m* and prior parameter *α*. In this study, we set *m* = 1.7 and ***α*** = 1. To visually display the clustering performance, we use four clustering performance indicators of accuracy, entropy, F-measure, and purity to show the clustering results. *R*=full_*t*_/block_*t*_ represents the ratio of the running time of the whole processing data set and the block processing data set of the algorithm, full_*t*_ represents the running time on the whole data set, and block_*t*_ represents the sum of the running time on each block. Although this part loads the data set into the memory at one time, this paper believes that *R* is similar to the data that cannot be loaded, because the total amount of data is the same, whether it is processed separately or at one time. Our experimental platform is AMD R5-5600X, six cores, 16G memory, Windows10 operating system, Matlab2016a.

### 4.2. Experimental Results on the Armstrong-2002-v2, Bhattacharjee-2001, and Heart Disease Data Set

To make SPFCM and OFCM algorithms run better, according to the suggestions of Havens et al. [25], we set the fuzzy index *m* = 1.7. For the Armstrong-2002-v2 data set, Bhattacharjee-2001 data set, and heart disease data set, the number of clusters is set to 3, 5, and 5, respectively. Because the sample size of these three data sets is small, they are not processed in blocks.  Table 1 shows the experimental results of the OFCM, SPFCM, and OWBFC algorithms. We can see that the OFCM algorithm and the SPFCM algorithm have similar clustering performances on these three different data sets, and it is difficult to compare the advantages and disadvantages of the two algorithms. But comparing the OFCM algorithm, SPCM algorithm, and OWBFC algorithm, it is easy to see that the OWBFC algorithm has the best clustering results except for some special cases.

### 4.3. Clustering Performance on DRD and HCV Data Set

Like the parameter setting in Section 4.2, the DRD and HCV data sets are divided into 5%, 10%, and 50% of the whole data set, and the last column of the HCV data set is selected as the basis for the number of clusters, the fuzzy index *m* = 1.7, and the number of clusters is set to 4. The OFCM, SPFCM, and OWBFC algorithms run independently 10 times on the basis of random initialization to calculate the maximum, minimum, and average values of accuracy, entropy, F-measure, and purity. The clustering results of the two data sets are shown in Tables 2–5. From Table 2, it can be seen that the accuracy of the OFCM is slightly lower than that of the SPFCM algorithm when the number of data blocks is large, and the accuracy of the OFCM algorithm is higher than that of the SPFCM algorithm when the number of blocks is small. Overall, the accuracy of OFCM algorithm is similar to that of SPFCM algorithm, and the accuracy of OWBFC algorithm is the best. Tables 2–5 show the accuracy, entropy, F-measure, and purity of these two different data sets. For example, 74.78/74.90/74.66 represents the mean, max, and min accuracy values, respectively. Compared with the OFCM algorithm and SPFCM algorithm, the OWBFC algorithm has the best results whether it is entropy or F-measure or purity. Because the OWBFC algorithm uses the MCMC sampling method to solve the parameters, it can obtain the global optimization of the parameters. Therefore, the OWBFC algorithm can obtain better clustering performance. Only from Tables 3–5, the gap between the three algorithms is not obvious. Combining with Table 8, it can be clearly seen that the OWBFC algorithm has good clustering performance and also greatly reduces the time consumption of the algorithm. Table 8 shows the running time at different division ratios. Because the data set name is too long, the abbreviation is used in the experiment.

### 4.4. Brain Images

Three brain images are shown in Figure 1. We use them to verify the clustering performance of OWBFC for large-scale image segmentation. We compare the OWBFC and BFC algorithms in this subsection. According to the recommendations [19, 25], the parameters *α* set to 1, and the parameters *m* set to 1.7. We split brain images at a ratio of 25% and set all classes to 3. Figures 2 and 3 show the clustering results of three brain images by BFC and OWBFC algorithms, respectively.  Table 6 shows the experimental results on three brain images.  Table 7 shows the running time results of BFC and OWBFC on three brain images. We can see from Table 6 that the clustering performance of OWBFC is better than that of BFC. Meanwhile, from Table 7, we can clearly see that OWBFC has a shorter time consumption compared with BFC. In summary, compared with BFC, the OWBFC algorithm not only maintains a good clustering effect but also consumes less time.

## 5. Conclusion

With the advancement of science and technology, the collection of various medical data has become more frequent and easier, which makes the scale of medical data larger and larger, and it is impossible to import the data into the memory at one time, so the hardware requirements for processing these data become higher and the time consumption increases. This paper proposes an OWBFC method, which reduces the memory consumption of the computer and the time consumption of the algorithm by introducing an online clustering framework to process the data set in blocks. From the experimental results, the block processing can effectively reduce the time consumption of the algorithm. However, the online clustering framework adopted in this paper needs to merge and save the cluster centers of each data block in the process of processing data, which raises the space consumption of the algorithm. Therefore, how to avoid excessive space consumption while ensuring low time consumption is a problem worth thinking about.

## Figures and Tables

**Figure 1:** Three brain images used in the experiment. (a) cta, (b) ctb, and (c) ctc.

**Figure 2:** Clustering results of BFC on three brain images. (a) cta, (b) ctb, and (c) ctc.

**Figure 3:** Clustering results of OWBFC on three brain images. (a) cta, (b) ctb, and (c) ctc.

**Algorithm 1:** Weighted Bayesian fuzzy clustering (WBFC) algorithm.

**Algorithm 2:** Online Weighted Bayesian Fuzzy Clustering (OWBFC) algorithm.

**Table 1:** Clustering performance on Armstrong-2002-v2, Bhattacharjee-2001, and Heart Disease data sets.

Data sets	Algorithms	Accuracy	Entropy	*F*-measure	Purity
*Armstrong-2002-v2*	OFCM	0.7235	0.4728	0.7948	0.7331
	SPFCM	0.7237	0.4697	**0.8011**	0.7372
	OWBFC	**0.7548**	**0.4632**	0.7964	**0.7489**

*Bhattacharjee-2001*	OFCM	0.8213	0.2879	0.8637	0.8235
	SPFCM	0.8635	0.2455	0.9294	0.8769
	OWBFC	**0.8792**	**0.2423**	**0.9328**	**0.8817**

*Heart Disease*	OFCM	0.7643	0.4675	0.7921	0.7039
	SPFCM	0.7659	0.4678	0.7914	0.7054
	OWBFC	**0.7768**	**0.4679**	**0.7932**	**0.7258**

The best average performances are shown in bold type in Tables 1–7.

**Table 2:** Accuracy (mean/max/min) on the DRD and HCV data sets (%).

DRD data set			
Block size	OFCM	SPFCM	OWBFC
5	73.16/73.32/72.95	73.26/73.37/73.18	**74.78**/**74.90**/**74.66**
10	73.34/74.44/73.12	73.37/73.54/73.15	**74.83**/**74.97**/**74.72**
50	73.53/73.64/73.31	73.51/73.62/73.43	**75.02**/**75.16**/**74.93**
HCV data set			
Block size	OFCM	SPFCM	OWBFC
5	74.16/74.41/74.11	74.17/74.31/74.09	**75.61**/**75.78**/**75.52**
10	74.29/74.44/74.16	74.24/74.42/74.13	**75.65**/**75.80**/**75.52**
50	74.37/74.48/74.31	74.33/74.47/74.25	**75.73**/**75.86**/**75.66**

**Table 3:** Entropy (mean/max/ min) on the DRD and HCV data sets (%).

DRD data set			
Block size	OFCM	SPFCM	OWBFC
5	47.72/47.88/47.65	47.77/47.92/47.61	**47.34**/**47.49**/**47.26**
10	47.75/47.89/47.67	47.77/47.91/47.63	**47.39**/**47.54**/**47.28**
50	47.81/47.95/47.76	47.82/47.97/47.74	**47.44**/**47.57**/**47.33**
HCV data set			
Block size	OFCM	SPFCM	OWBFC
5	46.65/46.78/46.52	46.79/46.87/46.68	**46.84**/**46.97**/**46.75**
10	46.69/46.78/46.53	46.81/46.89/46.72	**46.84**/**47.03**/**46.72**
50	46.71/46.82/46.66	46.88/46.96/46.75	**46.87**/**47.11**/**46.76**

**Table 4:** F-measure (mean/max/min) on the DRD and HCV data sets (%).

DRD data set			
Block size	OFCM	SPFCM	OWBFC
5	77.96/78.13/77.81	77.93/78.15/77.82	**78.42**/**78.57**/**78.30**
10	77.96/78.15/77.81	77.96/78.17/77.84	**78.47**/**78.60**/**78.33**
50	78.04/78.21/77.85	77.98/78.22/77.88	**78.51**/**78.63**/**78.38**
HCV data set			
Block size	OFCM	SPFCM	OWBFC
5	75.02/75.14/74.93	75.02/75.16/74.89	**75.96**/**76.13**/**75.84**
10	75.13/75.25/75.02	75.10/75.24/74.90	**76.03**/**76.17**/**75.91**
50	75.17/75.31/75.05	75.16/75.36/75.03	**76.15**/**76.31**/**76.02**

**Table 5:** Purity (mean/max/min) on the DRD and HCV data sets (%).

DRD data set			
Block size	OFCM	SPFCM	OWBFC
5	74.58/74.63/74.34	74.55/74.67/74.43	**75.27**/**75.43**/**75.16**
10	74.64/74.72/74.49	74.59/74.75/74.48	**75.31**/**75.46**/**75.24**
50	74.72/74.88/74.62	74.66/74.81/74.57	**75.37**/**75.50**/**75.26**
HCV data set			
Block size	OFCM	SPFCM	OWBFC
5	74.61/74.79/74.48	74.55/74.67/74.38	**75.25**/**75.37**/**75.18**
10	74.67/74.83/74.54	74.60/74.77/74.45	**75.29**/**75.43**/**75.16**
50	74.71/74.88/74.62	74.66/74.79/74.52	**75.33**/**75.46**/**75.19**

**Table 6:** Clustering results of BFC and OWBFC on three brain images (%).

Data sets	Methods	Accuracy	Entropy	*F*-measure	Purity
*Cta*	BFC	87.54	23.64	91.26	87.43
	OWBFC	**88.01**	**21.98**	**91.32**	**88.15**

*Ctb*	BFC	88.65	21.38	91.97	88.76
	OWBFC	**89.23**	**21.05**	**92.28**	**89.61**

*Ctc*	BFC	86.91	24.33	90.65	87.15
	OWBFC	**87.06**	**23.96**	**91.43**	**87.34**

**Table 7:** Running time on three brain images (s).

Image	BFC	OWBFC
Cta	1224.23	**345.36**
Ctb	1231.14	**339.45**
Ctc	1219.56	**326.72**

**Table 8:** OWBFC running time on different block ratios (s).

Data sets	Block size				*R*		
	100%	50%	10%	5%	100%/50%	100%/10%	100%/5%
DRD	85.31	67.54	15.67	12.51	1.26	5.44	6.82
HCV	97.25	70.26	17.48	13.16	1.38	5.56	7.38

## Data Availability

Armstrong-2002-v2 and Bhattacharjee-2001 data sets can be downloaded from https://schlieplab.org/Static/Supplements/CompCancer/datasets.htm. The other data sets can be downloaded from http://archive.ics.uci.edu/ml/index.php.
